# Modern Diagnostic Imaging Technique Applications and Risk Factors in the Medical Field: A Review

**DOI:** 10.1155/2022/5164970

**Published:** 2022-06-06

**Authors:** Shah Hussain, Iqra Mubeen, Niamat Ullah, Syed Shahab Ud Din Shah, Bakhtawar Abduljalil Khan, Muhammad Zahoor, Riaz Ullah, Farhat Ali Khan, Mujeeb A. Sultan

**Affiliations:** ^1^Department of Biochemistry, Faculty of Biological Sciences, Quaid-i-Azam University Islamabad, Pakistan; ^2^Department of Pharmacy, Faculty of Biological Sciences, University of Malakand, Pakistan; ^3^Women's Wellness and Research Center, Hamad Medical Corporation, Doha, Qatar; ^4^Department of Biochemistry, University of Malakand, Chakdara, Dir Lower, KPK, Pakistan; ^5^Department of Pharmacognosy, College of Pharmacy, King Saud University, Riyadh, Saudi Arabia; ^6^Department of Pharmacy, Shaheed Benazir Bhutto University, Sheringal, Dir Upper, KPK, Pakistan; ^7^Department of Pharmacy, Faculty of Medical Sciences, Aljanad University for Science and Technology, Taiz, Yemen

## Abstract

Medical imaging is the process of visual representation of different tissues and organs of the human body to monitor the normal and abnormal anatomy and physiology of the body. There are many medical imaging techniques used for this purpose such as X-ray, computed tomography (CT), positron emission tomography (PET), magnetic resonance imaging (MRI), single-photon emission computed tomography (SPECT), digital mammography, and diagnostic sonography. These advanced medical imaging techniques have many applications in the diagnosis of myocardial diseases, cancer of different tissues, neurological disorders, congenital heart disease, abdominal illnesses, complex bone fractures, and other serious medical conditions. There are benefits as well as some risks to every imaging technique. There are some steps for minimizing the radiation exposure risks from imaging techniques. Advance medical imaging modalities such as PET/CT hybrid, three-dimensional ultrasound computed tomography (3D USCT), and simultaneous PET/MRI give high resolution, better reliability, and safety to diagnose, treat, and manage complex patient abnormalities. These techniques ensure the production of new accurate imaging tools with improving resolution, sensitivity, and specificity. In the future, with mounting innovations and advancements in technology systems, the medical diagnostic field will become a field of regular measurement of various complex diseases and will provide healthcare solutions.

## 1. Introduction

Medical imaging is the process of visual representation of the structure and function of different tissues and organs of the human body for clinical purposes and medical science for detailed study of normal and abnormal anatomy and physiology of the body. Medical imaging techniques are used to show internal structures under the skin and bones, as well as to diagnose abnormalities and treat diseases [1]. Medical imaging has changed into healthcare science. It is an important part of biological imaging and includes radiology which uses the imaging technologies like X-ray radiography, X-ray computed tomography (CT), endoscopy, magnetic resonance imaging (MRI), magnetic resonance spectroscopy (MRS), positron emission tomography (PET), thermography, medical photography, electrical source imaging (ESI), digital mammography, tactile imaging, magnetic source imaging (MSI), medical optical imaging, single-photon emission computed tomography (SPECT), and ultrasonic and electrical impedance tomography (EIT) [2].

Imaging technologies play a vital role in the diagnosis of abnormalities and therapy, the refined process of visual representation which contributes to medical personnel access to awareness about their patient's situation [3, 4]. Electroencephalography (EEG), magnetoencephalography (MEG), and electrocardiography (ECG) are recording and measurement techniques that are not responsible to produce images, but these represent the data as a parameter graph *vs.* time or maps which shows the susceptible information with less accuracy. Therefore, these technologies can be said to form medical imaging on a limited scale. Worldwide, up until 2010, approximately 5 billion medical imaging techniques studies have been shown [5].

In the United States, approximately 50% of total ionizing radiation exposure is composed of radiation exposure from medical imaging [6]. Medical imaging technologies are used to measure illnesses, manage, treat, and prevent. Nowadays, imaging techniques have become a necessary tool to diagnose almost all major types of medical abnormalities and illnesses, such as trauma disease, many types of cancer diseases, cardiovascular diseases, neurological disorders, and many other medical conditions. Medical imaging techniques are used by highly trained technicians like medical specialists, from oncologists to internists [1].

Medical imaging technologies are mostly used for medical diagnoses. Medical diagnosis is the process of identification of patient disease and its symptoms. The medical diagnosis gives the information about the disease or condition needed for treatment that is collected from patient history and physical checkups or surveys. Due to no specificity of the many signs and symptoms of a disorder, its diagnosis becomes a challenging phase in medical science. For example, the case of erythema (redness of the skin) gives a sign of many diseases. Thus, there is a need for different diagnostic procedures the determination the causes of different diseases and their cure or prevention [7].

Historically, the first medical diagnosis composed by humans was dependent upon the observation of ancient doctors with their eyes, ears, and sometimes examination of human specimens. For example, the oldest methods were used to test on body fluids like urine and saliva (before 400 B.C). In ancient Egypt and Mesopotamia, doctors were able to measure the problem of the digestive tract, blood circulation, heartbeat, spleen, liver menstrual problems, etc. But unfortunately, medicine for curing diseases was only for wealthy and royal people.

At around 300 B.C., the use of the mind and senses as diagnostic tools was promoted by Hippocrates. He got a reputation as the “Father of Medicine.” Hippocrates supported a diagnostic protocol by testing the patient urine, observing the skin color, and listening to the lungs and other outward appearances. The link between disease and heredity also had been recorded by them [8]. In the Islamic world, Abu al-Qasim al-Zahrawi (Arabic physician) provided the first report on a hereditary genetic disease referred as hemophilia. In this report, he wrote about a family of Andalusia, whose males died due to hemophilia [9]. In the Middle Ages, many different techniques were used by physicians to detect the causes of imbalance function of the body. Uroscopy was the most common method of diagnosis. The patient's urine was collected in a special type of flask known as “Matula.” Urine was checked on the basis of color, smell, density, and presence of precipitate [10]. The viscosity and color of the blood were also examined by physicians to detect chronic or acute diseases [11]. The pulse rate, power, and tempo of a patient's artery were observed by physicians through a technique known as palpation [12]. In Middle Ages, physicians were also used to combining the study of medicine and zodiac signs [13].

In the 19^th^ century, X-rays and microscopes were the diagnostic tools that helped to diagnose and treat illnesses. At the beginning of the 19^th^ century, medical doctors diagnosed diseases by the examination of symptoms and signs. By the 1850s, many diagnostic tools such as ophthalmoscopes, stethoscopes, and laryngoscopes lead to evoke the medical doctors with the sensory power to develop other novel methods and techniques for diagnosing different illnesses. And in this way, a series of diagnostic tools including chemical tests, bacteriological tests, microscopic tests, X-ray tests, and many other medical tests were generated [8].

Medical imaging techniques are developed after the discovery of X-rays. In November 1895, Wilhelm Conrad Roentgen discovered X-ray. He got the Nobel Prize in 1901 for his discovery. Radiologists gave names to X-ray basis as “X-rays” or “plane film” used for diagnosing bone fractures and chest abnormalities. Fluoroscopy was developed due to a more powerful beam of X-ray for diagnosing the patient abnormalities. In 1920s, radiologists started giving information about various diseases like cancer of the esophagus, ulcers, and stomach. Fluoroscopy is now converted into computed tomography (CT).

Today CT scan is commonly used to diagnose many diseases. The mammography technique also uses an X-ray beam, to generate high-resolution breast images, monitoring breast cancer. In the 1940s, the X-ray tomography technique was developed, looking for a desired part of the tissue. In this technique, the whole process was accomplished by rotating the tube of X-ray focus on part of the tissue. Today, tomography is replaced with advanced imaging techniques such as CT scanning or computerized axial tomography (CAT) scanning. X-ray is also a source of a technique known as “angiography,” which is used to obtain images of blood vessels. In 1950s, diagnostic imaging tests along with nuclear medicine were started. Radioactive compounds are used as X-ray sources rather than X-ray tubes. Radioactive compounds produce gamma rays. They are joined with other complexes that are an essential part of the disease analysis to study a certain illness. For an instant, technetium 99m is combined with methylene diphosphonate, which is absorbed by bone tumors. In this way, breast or lung cancer spread to other body parts such as bone can be detected from this type of nuclear bone scan technique [14].

## 2. Advance Modalities in Medical Imaging

Many advanced techniques are developed and can be explained with their principle of work, application in medical labs, and development in imaging techniques. Computed tomography (CT), positron emission tomography (PET), magnetic resonance imaging (MRI), single-photon emission computed tomography (SPECT), digital mammography, and sonography are included in advanced medical imaging techniques. These are all mentioned below to understand their advantages and applications in the diagnosis, management, and treatment of different diseases such as cardiovascular disease, cancer, neurological illnesses, and trauma. These techniques are readily used by clinicians because through images, they can easily choose how to manage diseases.

## 3. Computed Tomography (CT)

In the 1969s, Hounsfield invented the first CT-scanner prototype [15]. Computed tomography is also known as X-ray CT. A CT scan is used by radiologists, biologists, archaeologists, and many other scientists to generate cross-sectional images of different scanned objects. A modern CT scanner system is shown in Figure 1. In the medical field, technicians use CT scanners, machines to produce the images that lead to diagnosing the abnormalities and other therapeutic measurements. In this technology, X-rays are produced from different angles that are eventually processed by computers to create tomographic images. This computer-based technology has been greatly improved, developing reconstructed images with high revolution [16]. In the pharmaceutical industry, it has been used to study and improve the medicine manufacturing process to generate good quality products [17].

Positron emission tomography (PET) and single-photon emission computed tomography (SPECT) are the types of CT scan. An X-ray generator is used to generate the X-rays that rotate nearby the object to be scanned. X-rays are detected by an X-ray detector located on the opposite side of the source of X-rays. A sonogram is obtained, which is a visual representation of raw form data. This scanned data is processed in the form of tomographic reconstruction that leads to generating a series of cross-sectional photos. CT scan is performed by special individuals called radiology technologists or radiographers. Over the last two decades, CT is used largely in many clinical labs in different countries [18]. According to an estimated study, almost a 72 million scans were achieved in the US in 2007 and 80 million scans in 2015 [19].

CT is an effective technique for monitoring various types of cancers such as cancer of the bladder, kidneys, skeleton, neck, and head and for diagnosing infection [20–22]. CT also identifies distant metastases to the lungs, skeleton, liver, and brain. CT has made a high impact on the brain and lungs [23, 24]. CT scan is the best method than other techniques in detection as well as recording modifications in tumor mass during treatment [25]. It may show a bloated belly with enlarged lymph nodes in patients with bronchus carcinoma. In this way, CT scan help in performing before surgery [26]. Another major application of CT scans is the detection of heart diseases like myocardial disease, congenital heart disease, and coronary artery bypass grafts [27]. Gastroenterologists mostly use computed tomography for the analysis of the liver or pancreas of patients. Tumors of size 1.5-2.0 cm in diameter can be detected by CT scan. Furthermore, biliary obstruction caused by lesions can also be monitored by this technology [28]. One of the rewarding roles of technology is to study suspected intra-abdominal abnormalities with 95% accuracy, and treatment decisions can be easily made [29].

A big drawback of computed tomography is that large masses within the gastrointestinal tract may not be visible during the abdominal investigation. There is also no finding of some of the mucosal abnormalities by it. CT scan is highly useful to manage abdominal disorders such as carcinoma of the stomach, esophagus, and rectum more accurately as compared to other modalities [30, 31] The middle column of the spine can be visualized by using the computed tomography technique during dislocation type of fractures in many thoracolumbar fractures. CT also detects lesions and provides nonsurgical management of some disorders, for example, unstable burst damages [31].

All spinal injuries are unstable and known as translational injuries. Before surgery of such patients, complete information about the site of ligament discontinuity of respective vertebrae is provided by computed tomography. It also gives the prediction of whether Harrington-rod stabilization is possible or not. CT scan can provide detailed evidence of distraction injuries and fractures. For example, flexion-distraction injury between the 11^th^ and 12^th^ thoracic vertebrae and spinal injury between the 2^nd^ and 3^rd^ lumbar vertebrae have been scanned by computed tomography scan as shown in Figures 2 and 3, respectively [32].

Advanced CT bone imaging techniques include volumetric quantitative CT (QCT), high-resolution CT (CT), and micro-CT. High-resolution CT and high-resolution MR are generally used *in vivo*; micro-CT and micro-MR are usually used *in vitro* systems. These advanced modalities are used for bone imaging to investigate bone diseases especially osteoporosis and bone cancer. In osteoporosis, disorder advanced CT bone imaging provides information about bone mineral density (BMD), bone strength, a risk factor for osteoporosis, and recovery factors after medication or bone therapy.

Dual-energy X-ray absorptiometry (DXA) and volumetric QCT are the quantitative methods used for weighing the macrostructure of suspected bone. High-resolution CT and micro-CT methods are applicable for measuring the microstructure of trabecular bone without any invasiveness or destructiveness. CT and MRI have been used to obtain bone structure. However, the CT field has been more developed as compared to other techniques, because there are more advantages of CT-based modalities; for example, QCT generates three-dimensional (3D) images in such a way that trabecular and cortical bone can be distinctly measured. vQCT technology is quicker than MRI [33].

## 4. Volumetric Quantitative CT (vQCT)

Initially, QCT has been used to measure trabecular BMD of the forearm and lumber midvertebrae through a particular transverse CT slice. The measurement of BMD is a static property of the advanced spiral QCT [34]. Trabecular bone in the spine and cortical bone in the hip may be indicated by this technology to estimate the fracture risk [35].

For the improvement of the 3D structure of the cortex, almost 0.5 mm isotropic spatial resolution is required, but still, almost 1.5 to 2 mm resolution is provided by QCT which is not adequate to make accurate images. This is a drawback of QCT. In general, the measurement of accurate cortical thickness for the femur is easier than the thickness in the spine, especially in aged people. Researchers have shown that women grow faster not only with small vertebrae as well as reduced bone mass but also with a slow rate of increase in cross-sectional area as compared to men [35]. QCT is a CT imaging technique that can provide information about bone density. For example, a QCT scan of the femur for the measurement of macrostructure and bone mineral density (BMD) has been shown in Figure 4(a) [33].

## 5. High-Resolution CT (hrCT)

High-resolution CT is a modern CT scanner that usually requires a high radiation dose but produces high-resolution images of bone such as forearm bone submitted to CT to determine the trabecular and cortical network and texture as shown in Figure 4(b) [33]. According to many different cross-sectional studies, CT gave better imaging results in distinguishing fractured vertebral trabecular structures from nonfractured structures as compared to DXA measurements of BMD [36].

## 6. Micro-CT (*μ*CT)

Micro-CT with 1-100 *μ*m spatial resolution is typically known as microscopy. Micro-CT has abilities to replace the standing techniques used in in vivo measurements in rats and mice like animals. Initially, the micro-CT technique used synchrotron radiations to obtain ultra-high-resolution applications [37].

Mostly, now, the convenient method of X-ray tube-based micro-CT is used in university-based research laboratories and special clinical centers. To make 3D structures of bone, some special software (for example, FEM) is attached with a micro-CT scanner. Finite element modeling (FEM) is a software mostly used in engineering. Its goal is to help information of 3D structures of bone for analysis of fractured bone part structures from nonfractured bone structures. Currently, structural models are generated by volumetric QCT, and computer-based programs give the element elastic properties from the bone density at the site of elements [38].

Arlot and coworkers determined the 3D microstructure of bone of postmenopausal women with osteoporotic disease; they have accomplished treatment with proper strontium ranelate therapy for 36 months [39]. Researchers investigate these 3D micro-bone structures as shown in Figure 5 [33]. Over the past two decades, considerable development occurred in imaging technologies for osteoporosis bone disease analysis. Despite the development in these technologies, there are many challenges for bone imaging, such as the sample size, spatial resolution, complexity, radiation exposure, time, and cost. Finally, there is still a requirement of high accuracy, availability, reproducibility, and proper monitoring procedure for better bone imaging [33].

CT scan for lung disease is highly used in present days. For example, a low-radiation helical chest CT scan is used to investigate lung cancer (bronchopulmonary cancer) [40, 41]. Another lung disease is the most common type of progressive idiopathic interstitial pneumonia mostly in adults known as idiopathic pulmonary fibrosis (IPF). In IPF patients, CT-based methods include density histogram analysis, CT scan of whole lungs, and density mask technique, and other structural or texture classification methods are greatly used to examine the pulmonary function, lung disease progression, and mortality. For example, lung images of a 73-year-old male IPF patient have been taken by CT as shown in Figure 6. These methods have the property of time efficiency, availability, and reproducibility. Still, there are many issues interrelated to computer-based CT in IPF disease analysis. But it is promising by scientists to develop advanced CT imaging techniques that must play a vital role in the future to manage lung diseases as well as other abdominal diseases [42, 43].

There are many possible reasons for the usage of CT scans, for example, to determine or investigate the acute stroke in the patient's head. CT is applicable to establish the diagnosis, investigate the type of stroke, respond to surgery, and finally manage the disease [44]. CT scan of the head is also responsible for the investigation of dementia disease. Accurate diagnosis is directly related to proper management of symptoms and signs of dementia. Patients with treatable lesions can also be identified by computed tomography [45]. Abdominal computed tomography is a new technology for identifying fungal infection known as disseminated fungal infection (DFI) in pediatric cancer patients. Currently, abdominal CT is greatly applicable for the diagnosis and management of DFI in cancer patients [46]. During the past few years, the usage of CT scan has become a national trend in emergency departments, especially in the US. Computed tomography plays an expanding role in diagnosing acute and chronic diseases as well as life-threatening diseases such as stroke, head injury, major trauma, heart disease, abdominal pain, pulmonary embolism, severe chest pain, and renal abnormalities [47].

## 7. 3D Ultrasound Computed Tomography (3D USCT)

3D USCT is a promising technology for imaging breast cancer. Simultaneous recording of reproducible reflection, speed of sound volume, fast data collection, attenuation, and high image quality production are all the main advantages of the USCT system. 3D USCT system is a full potential device used for clinical purposes. Only in 4 minutes, the full volume of breast can be picked up [48].

## 8. Risks of Computed Tomography

Computed tomography risks are small but if these small risk**s** are produced by million numbers of scans, they may drive into serious public health concerns in the future, especially from pediatric CT. The risk of cancer due to computed tomography scanning is increasing [49]. Children are of specific concern due to the sensitivity of radiation-induced cancer as compared to adults. According to a study, the risks of leukemia and brain tumors are mostly revealed after exposure to radiation from CT scans [50].

According to the authors of a recent report “long-term risks from CT scans directly would require very large-scale studies with lifelong follow-up.” The author gave this statement after the study date on CT scan exposure leading to the risk of future cancer [51]. Radiologists should be a source of discussion earlier to perform imaging technologies that contain high doses of radiation. They should also know about the risk factors of imaging technologies that can cause more adverse effects than recovery. Both families and patients should also raise the question/answers about the benefits and risks of CT scans [52].

## 9. Positron Emission Tomography (PET)

Positron emission tomography is a nuclear medicine functional technique that is used to display the total concentration of radioactive labeled elements in the body with clear images. It has the potential to diagnose biological processes within living bodies and is highly applicable for clinical purposes [53]. 3D images of positron-emitting radionuclides within the body are made by a computer system. In PET-CT scanners, 3D imaging is created with the help of a CT X-ray scan implemented on the patient body in the same machine and session. Positron emission tomography (PET) and nuclear magnetic resonance (NMR) both are quantitative radiological techniques that display information about biochemistry and physiology, normality, or abnormality. Nuclear magnetic resonance is not more sensitive to give high-resolution images by the distribution of substances except hydrogen. It can measure the total concentration of ATP and creatine phosphate (CP) in particular areas of the brain. Thus, both NMR and PET performed their specific function in the diagnosis. In 1953, the first PET system was established at Massachusetts General Hospital. It was followed by many other devices in a series manner such as tomographic positron camera, PET scanner, and other PET instruments [54].

## 10. Working Principle of PET

The PET technique detects radioactivity emission when a small concentration of radioactive tracer is intravenously injected. These tracers are frequently labeled with carbon-11, nitrogen-13, oxygen-15, and fluorine-18, as shown in Figure 7. There is no positron emitter of hydrogen. The radioactive dose amount is the same as used in CT. 10-40 minutes is required to complete the process to perform a PET scan. The patient is fully clothed during scanning. There are specific steps in PET scan processing, explained in Figure 7 [55].

Two molecular probes are mostly used to explain PET assay: 2-[F-18] fluoro-2-deoxy-D-glucose (FDG) and 3-deoxy-3-[F-18] fluorothymidine (FLT). FDG is the analog of F-18-labeled glucose, and it is used to identify diseases by changing the metabolism of glucose in heart diseases, Alzheimer's disease, and cancer. FLT is the analog of F-18 labeled thymidine and is highly used to estimate processes like cell proliferation and DNA replication by analysis of the phosphorylation process and thymidine transport. Thus, FLT and FDG are considered as best candidate probes/tracers for molecular imaging.

An early diagnosis of Alzheimer's disease can be scanned by PET technology with 93% accuracy. Huntington's disease, a hereditary disease was also detectable by PET scan. The development of PET technology provides accurate whole-body images for examining early primary and metastatic diseases. Imaging of transgenes provides information on the regulation of gene expression during cell proliferation, growth, response to environmental stimuli, the aging process, and gene therapy. Such endogenous gene expression can be monitored through the developed PET approach, which uses F-18-labeled oligodeoxynucleotides having a short single strand of almost fifteen nucleotides. In monkeys with 1-methyl-4-phenyl-1,2,3,6-tetrahydropyridine- (MPTP-) induced lesions on one side of the brain, the study of restoring dopamine production by gene therapy can be assessed by PET imaging, as shown in Figure 8 [56].

The combination of PET and computed tomography (PET-CT) forms a hybrid imaging approach that is highly used to gain functional and metabolic information to measure inflammatory and infectious diseases to assess their proper treatment. PET-CT hybrid imaging technique can provide quick information during the diagnosis of a disease and its treatment response [57].

Haberkorn et al. measured FDG uptake that relates to the proliferation rate of tumor cells in the head and neck with different patterns, in two groups of patients [58]. The FDG uptake was also measured in the malignant neck and head tumors and metastases process by the use of FDG-PET. Minn and coworkers found that the uptake of FDG is related to the proliferation rate of tumor cells [59]. Jabour *et al.* measured the normal anatomy of the neck and head [60]. In this way, change in uptake FDG as investigated by PET provides necessary information for clinical and anticancer therapeutics [61].

In the human cerebellum, changes in local neuronal function by voluntary movement and tactile stimulation were also mapped with the help of the PET approach detection of brain blood flow. According to research, finger movement leads to the production of parasagittal and bilateral blood flow enhancement in the superior and anterior hemispheric cortex of the brain human brain cerebellum. The enhancement in midline blood flow in the posterior vermis of the human brain cerebellum is produced by saccadic eye movement. PET also allows the measurement of structural and functional relations in the cerebellum of the human brain [62]. The development of the PET brain imaging technology makes it possible to advance understanding of the anatomy of brain parts and map of neuroanatomical basis of cognitive processes and memory [63]. A pathogen SIV (simian immunodeficiency virus) causes infection in rhesus macaques (a type of monkeys) with acute viremia, and progression leads to infection in the solid tissues of lymphoid, and then, cellular degradation becomes a terminal disease, and death occurs in most cases. So, the FDG-PET imaging technique is used to take images from SIV-infected animals. In this way, infected groups can be distinguished from the uninfected control groups [64].

## 11. Future of PET Technology

The PET scan can be used to measure the concentration of amino acids, sugar, fatty acids, and receptor in the living body. It is a new diagnostic tool used to detect diseases such as atherosclerosis, aging, cancer, and schizophrenia, although improvement in instrumentation and modeling is still required for future purposes. Emission tomography has also been associated with a small risk of ionizing radiations [54].

## 12. Magnetic Resonance Imaging (MRI)

Magnetic resonance imaging (MRI) is primarily an imaging technique that is applicable for noninvasive visualization of the anatomy and physiology of the body in both disease and health conditions. An MRI-related technique known as echo-planar imaging (EPI) was developed by physicists Peter Mansfield and Paul Lauterbur in the late 1970s [65]. Magnetic fields, electric fields, and radio waves are used in an MRI scanner to produce images of organs and the structure of the body. The SI unit of magnetic flux density (magnetic field strength) is measured in tesla (T).

The most common detections by MRI are multiple sclerosis, CNS tumors, brain and spine infections, stroke, injuries in ligaments and tendons, muscle degradation, bone tumor, and occlusion of blood vessels. MRI uses nonionizing radiation, frequently preferable compared to CT. MRI also provides excellent contrast of soft tissues; for example, the white and gray matter structure of the brain can easily be distinguished through this approach. MRI employs other different techniques such as functional MRI, magnetic resonance angiography (MRA), susceptibility-weighted, diffusion-weighted (PWI), diffusion-weighted (DWI), gradient echo, and spin-echo. It provides an image of good quality without requiring repositioning of the patient [66]. There are several benefits to MRI such as it is a painless, noninvasive technique with high spatial resolution and nonionizing radiations. MRI is mostly used independently for soft tissue analysis.

## 13. Working Principle of MRI

An MRI machine consists of multiple components, including a slab for patients to lie on, a superconducting magnet, a protective cage, the operator's console, and computers to analyze the data and product images. During the MRI scanning process, the machine's magnet produces a strong magnetic field. Hydrogen ions align in the target body part of the patient due to a stable magnetic field. Then, bombardment of radiofrequency waves causes the alignment of lined-up hydrogen ions to move out, and then, ions return to their equilibrium state [67]. An attached computer system converts the spin echoes (signal) of hydrogen ions into the images, after several “shifting” and “working on.” A microphone is also present inside the MRI unit for communication between the patient and technologist during the imaging process. Images of only the target part of the body are created through MRI radiological analysis. The physician chooses which part of the patient's body must be analyzed by imaging, to diagnose the illness of the patient [68].

## 14. Applications of MRI

A major application of whole-body MRI is to investigate skeletal metastases. The MRI approach allows for visualization of the tumor because the tumor matrix contains an abundance of the proton. It is a more sensitive imaging technique than skeletal scintigraphy (bone scan) in the measurement of skeletal metastases. The whole-body MRI technique is more effective for detecting lesions in the pelvis, spine, and femur. This technique is also highly used as a primary diagnostic tool for the measurement of soft tissue diseases, whole-body fat, and polymyositis disease [69].

MRI is different from other diagnostic techniques because MRI has no risk of ionizing radiation. MRI has no side effects unlike CT and PET scans. There is no loss of image quality due to the scanning of body target parts from several angles and viewpoints [70]. Dynamic contrast-enhanced magnetic resonance (DCE-MRI) has been developed for the detection of the tumor microenvironment and its treatment. It has been supported as a useful method and improved clinical interest [71].

An advantage of using MRI to diagnose cardiovascular diseases is that examination reveals function structure perfusion, metabolism, and blood flow in the heart. A cardiovascular MRI is a source for the detection of congenital cardiac diseases, abnormalities in the thoracic aorta, and pericardium in heart patients. During the detection of myocardial tumor or right ventricular dysplasia, tissues are differentiated due to varying imaging parameters of the MRI approach. Another application of MRI, cardiovascular MRI, is applicable for determining cardiac prognosis, ischemia in a patient with heart disease, artery arteriosclerosis, and screening the myocardial viability [72].

Schizophrenia patients show mental abnormality which leads to language processing deficits and abnormal social behavior. Functional MRI has been applicable for remarks of such types of illnesses. The region of hypoactivity can be determined in the frontotemporal cortex of the patient brain. Soft neurological signs and symptoms have also been promoted. Functional MRI can detect abnormalities in the cerebrum; cerebral asymmetry images reveal changes in patients with schizophrenia compared with control as shown in Figure 9 [73].

Microfluidic LOC (lab-on-a-chip) is a device used as an emerging technology in medical laboratories. Sample (consist of suspensions of cells) and reagents react on these devices. For monitoring reaction on LOC, MRI is considered an ideal tool. MRI records the signals from the expended fluid leavings in the device. MRI combined with MRS (magnetic resonance spectroscopy) monitors fluid flow processes, chemical reaction separations, and diffusion processes in LOC. But MRI and MRS both show low sensitivity. In the future, there is a hope that MRI will be applicable for the advancement of microfluidic LOCs with powerful usage in medical diagnostic libraries [74].

Mutation in BRCA1 and BRCA2 genes leads to losing their ability to repair the damaged DNA, causing cancer, especially breast cancer. MRI diagnoses breast cancer which is due to a genetic mutation. Mostly, these hidden breast cancers are not detected by mammography. For a decade, doctors use MRI imaging tools to detect breast cancer [75]. According to previous research, 27-37% of patients have shown lesions on MRI, which are not seen through mammography. The researchers noted that mammography had a low value of positive prediction of 52.8%, as compared to MRI which is high at 72.4% [74].

Molecular MRI employed for specific and early detection of pulmonary metastatic cancer cells can improve its treatment. In research, pulmonary cancer cells are besieged by iron oxide nanoparticles having the ability to bind with ligand expressed on the cells. Then, images were taken by high-resolution hyperpolarized ^3^He MRI (HP ^3^He MRI). The study confirmed that HP ^3^He MRI pooled with targeted superparamagnetic iron oxide nanoparticle (SPION) contrast agent detects specific and early metastatic pulmonary cancer in mice. A researcher used the LHRH-SPION agent to explore new drug procedures. For this purpose, they injected breast adenocarcinoma cells into mice and then detect pulmonary defects as cancer formation in mouse lungs with the help of LHRH-SPIONs and HP ^3^He MRI results are shown in Figure 10 [76].

Multinuclear 3D solid-state MRI allows images of tooth bone and calcium phosphate components of bone substances. It also gives information on the bone composition and texture of the bone [77]. Recent neuroimaging techniques including high-resolution MRI can investigate myeloarchitectural patterns in the cortex of the human brain. The bands of myelination have been revealed by the staining technique. Now, the same band in good quality image form can also be obtained by high-resolution MRI imaging technique. Although the advanced technology has been largely applied in the visual system, further improved methodologies are required for the investigation of another brain region. To overcome high ratio of “signal” to “noise” is a challenge for MRI machines that is produced due to the increased resolution of the image [78]. In this way, fMRI and other types of MRI have been powerfully used to change our understanding of diseases, their causes, and how to manage the conditions.

## 15. Simultaneous Imaging with MRI and PET

In *in vivo* study, imaging of small animals, for example, mouse imaging by combined MRI and PET modalities, produces constant information of different parts of the body. An experimental study reveals that the combined PET/MRI technique improves the understanding of malignant tissues and heterogeneous tumors, edema, and necrosis that are not done by MRI alone. Particular ionic ^18^F is also used for PET/MRI combined imaging of small animals as models of bone metastasis, osteoporosis, and arthritis to study the complete skeletal system [79].

## 16. Risks of Magnetic Resonance Imaging

Magnetic resonance imaging (MRI) is highly expensive, low in sensitivity, and time-consuming for scanning and processing compared to other imaging modalities. A probe with a bulk quantity may be needed for MRI. It cannot detect abnormalities of intraluminal body parts. It gives no real-time information. And it can create a suffocating environment for some people [2].

## 17. Single-Photon Emission Computed Tomography (SPECT)

Single-photon emission computed tomography (SPECT) is an advanced imaging technique using gamma rays and provides three-dimensional (3D) representations of objects with high accuracy. In 1963, Kuhl and Edwards [80] gave the first report about single positron emission computed tomography. Gradually, modification with new instruments such as computer-attached systems and rotating gamma cameras leads to the development of a novel modality of single-photon emission tomography.

SPECT has become a great medical imaging technique used in research and clinical area. A dual-headed single-photon emission tomography (SPECT) system has been shown in Figure 11 [81]. It monitors the 3D information of an object by producing series of thin slices from tomographic images. These essential tomographic images can improve the ability detection of deep and very small fractures in patients [81].

SPECT assesses the multiple two-dimensional (2D) images from different angles by using high-energy gamma rays. Data is reconstructed and recorded, and 3D images of the target portion of the body are produced by a computer program. SPECT is greatly used in clinics and research laboratories like other tomographic modalities such as PET, MRI, and CT. SPECT and PET both use the radioactive tracer and then measure the emitted gamma rays. In the case of SPECT, emitted gamma rays by radioactive tracers are directly detected by the detector. The computer system analyzes the data from the detector and produces the true image of the area where the radioactive tracers are injected. SPECT imaging technique is less expensive than exclusively used for imaging small animals. It is sensitive to monitoring target bone metabolism, myocardial disorders, and blood flow in the cerebrum [82].

SPECT has also been designed for imaging of the brain known as neurochemical brain imaging. It has a powerful imaging technique to elaborate the neuropsychiatric diseases. It is an essential developmental technique that has great potential to monitor the pathophysiology and many other complex disorders of the brain [83].

Today, hybrid SPECT and CT are progressively employed and available in the nuclear medicine field. SPECT/CT provides exact abnormal bone turnover during inflammation, bone tumor, bone regeneration, bone infection, and trauma in complex bone joints such as the knee, hip, foot, shoulder, and hand/wrist. In most cases, CT with specificity and SPECT with high sensitivity are performed together for a complete diagnosis. SPECT/CT is also responsible for giving the proper information about therapy planning. For example, it tells us about the decision of using SPECT/CT alone or joint arthroplasty. It was observed that joint arthrography of the knee gives better results as compared to SPECT/CT alone as shown in Figure 12 [84].

SPECT/CT technique has great potential for the measurement of articular cartilage, soft bodies, and synovial structures. It also gives promising results in the examination of osteochondral abnormalities [84].

## 18. Risks of Single-Photon Emission Computed Tomography (SPECT)

Single-photon emission computed tomography (SPECT) is expensive and requires additional care for performance with radioactive materials. Like PET, it uses ionizing radiation and creates radiation side effect for the patients [2].

## 19. Digital Mammography

Mammography is a technique used to screen and diagnose human breasts. Low-energy X-rays (30 kVp) are used in the mammography in performing early diagnosis and screening of human breast cancer. Ionizing radiations are used in mammograms to create images for analysis of abnormal conditions. Ultrasound is usually employed to give additional information about masses, detected by mammography. MRI, discography, and positron emission mammography (PEM) are also supporters of mammography. Mammography is more accurate for women 50 or above 50 years old as compared to younger women because old women have high breast density [85]. Today, conventional mammography has been replaced by digital mammography.

An advanced technique is used for creating 3D images of breast tissues for detailed analysis of breast cancer, known as 3D mammography. When 3D mammography is used along with usual mammography, it gives more positive results [86]. Cost-effectiveness and high radiation exposure are of high concern to 3D mammography [87].

Digital mammography is a special form of mammography employed to investigate breast tissues for breast tumor study. Digital mammography contrasts with film (conventional) mammography by using a special detector that detects the transmitted X-rays energy and converts it into an image signal by a computer system instead of a film X-ray. Digital mammography is a rapid and advanced modality that has the potential for diagnosis and proper screening of breast cancer. Such new diffusion technologies can alter the health care pattern through many mechanisms. There are different results related to breast health care for digital-screen and film mammography. Digital mammography may also change the application of diagnostic services ensuring mammograms with positive screening [88].

Digital mammography has been considered a better technique as compared to film mammography in the detection of breast cancer in premenopausal, premenopausal, and young women. A digital system has more cost (approximately 1.5 to 4 times) than a film system. Digital mammography has the advantage of diagnosis in computer-based system that generates images with easy access and better-quality transmission, recovery, and image storage. Advanced digital mammography uses an average low dose of radiation without cooperation with diagnostic accuracy [89].

A healthy breast tissue mammogram recorded by digital mammography is clear as compared to a mammogram on film as shown in Figure 13 [90]. Scientists used both digital mammography and film mammography for 42,760 women's breast X-rays. Cancer is almost equally well detected through these techniques. But digital mammography detected 28% more breast cancer in younger women or those under 50, who have dense breast tissues. Digital mammography uses a specific detector that captures the transmitted X-rays and sends the information in the form of energy that converts into an image through a computer system [90]. Digital mammography screening for breast cancer is not cost-effective, relative to conventional mammography [91].

Now, screening MRI is highly used as an adjunct to mammography, recommended for women to ensure 20-25% or more threat of breast cancer [92]. Currently, breast cancer diagnostic programs have been recognized widely at least in 22 countries. Collective struggles lead to the formation of the Breast Cancer Screening Network (IBSN), an international program for policymaking, administration, funding, and handling of results that come from breast cancer screening of huge populations [93]. The ultrasound technology combined with mammography is used to detect elevated risk factors for breast cancer. According to research on elevated risk factors, by using ultrasound with mammography, more than 90% of cancer risk was seen in over 50% of women having dense breast tissues, and 25% of cancer risk factors were determined in women having just 26%-40% dense tissues of the breast. It is suggested that screening with ultrasound may be beneficial for those women having other risk factors and less dense breast tissues [94].

## 20. Medical Ultrasound

The ultrasound imaging technology was used earlier as a diagnostic tool for brain images. Today, ultrasound is a widespread imaging technology used in diagnostic laboratories and clinics. It is free from radiation exposure risk, comparatively less expensive, and highly portable as compared to other imaging techniques like MRI and CT [95]. This system is used in different fields. In the medical field, ultrasound uses sound waves of high frequency, to diagnose the organs and structure of the body. The ultrasound system is performed with high frequency. Special technicians or doctors use it to observe the kidney, heart, liver, blood vessels, and other organs of the body. The most critical component of ultrasound is a transducer. An ultrasound transducer can convert an electrical signal into sound waves and sound waves into an electrical signal. An ultrasonic image or sonogram is formed by transmitting pulses of sound waves into tissues using a special probe. Different tissues reflect these sounds to a different degree. These reflected sound waves (echoes) are detected and presented as an image with the help of the operator. In the medical field, there are many applications of ultrasound. Ultrasound scanning is a very effective and reliable technique that is greatly used for monitoring normal pregnancy, placenta previa, multiple pregnancies, and different abnormalities during pregnancy and rest [96].

An ultrasound imaging technique also known as transvaginal ultrasound (TVS) alters our understanding of the management and diagnosis of pregnancy. The TVS gives clear knowledge of early pregnancy problems. It investigates the pregnancy location as well as viability. *In utero*, the TVs have determined the fetal heart activity that is initial proof of pregnancy viability. Abnormal development in fetal heart rate pattern indicates the subsequent miscarriage. Less fetal heart rate especially at 6 to 8 weeks demonstrates subsequent fetal disease. Fetal heart pulsation can be seen on TVS. The routine use of TVS also leads to development in managing early pregnancy failure. Awareness of pregnant women and improvement in early pregnancy units can directly manage miscarriage. TVS is a very sensitive approach for diagnosing early miscarriage. It detects trophoblastic tissue and blood flow in the intervillous space, and the use of color Doppler images leads to estimate the level of expectant management [97].

Functional ultrasound (fUS) is highly applicable for imaging the brain and detects transient alternation of blood volume in the brain at high resolution than other brain imaging modalities. The blood volume in small vessels can be measured by functional ultrasound (fUS), which uses plane-wave illumination with a high frame rate. Functional ultrasound can detect the brain's active portion [98]. Ultrasound has major advantages as noninvasive and out-patient scanning in children to investigate neuromuscular disorders. Ultrasonography has been used for finding the normal function of muscle, muscle contraction, muscle thickness, and muscle fiber length. Real-time ultrasound is used for muscle imaging. When ultrasound applies to neuromuscular patients, different muscle disorders can be detected by a pattern of muscle echo, such as a bright spotted pattern of increase in muscle echo obtained in muscular dystrophy patients and a moderate increase in echo showed in spinal muscular atrophy [99].

Currently, early care physicians can easily understand complex patient conditions with the help of advanced 3D ultrasound algorithms. And high-speed networks are used in special health centers to enhance patient care facilities [100]. 3D ultrasound is widely used due to the reason of 2D ultrasound limitations. Clinical 3D ultrasound experience has an advantage in the diagnosis of disorders and produces a 3D image that guides invasive therapy. Further improvement in 3D imaging software, as well as hardware, will lead to routine usage of this tool [101].

High-resolution ultrasound which is also known as ultrasound biomicroscopy (UBM) has clinical applications in imaging the human eye. UBM uses 35 MHz or above frequencies to provide images of high resolution as compared to conventional ophthalmic ultrasound techniques. UBM can be used to diagnose ocular trauma and complex hypotony. It can determine eye lens displacement, iridodialysis, zonular flaw, cataract, lens subluxation, and hyphemia. Hyphemia is a condition in which blood diffuses the anterior chamber of the eye due to injury. Hyphemia scan image by Sonomed UBM is shown in Figure 14 [102].

UBM can detect several eye abnormalities, as it allows for the diagnosis of trauma, glaucoma, and foreign bodies. It can evaluate eyelids, neoplasms, normal eye anatomy, and extraocular muscles during strabismus surgery. Currently, for high-resolution diagnostic eye imaging, new advanced technologies such as pulse encoding, transducer array, and ultrasound combination with light are developed [102].

A high-frequency (40 MHz) ultrasound imaging technique has been developed for checking the programmed cell death process known as apoptosis. It is a noninvasive procedure used to monitor the apoptosis process that happens because of agents especially anticancer agents in cells of body tissue in vitro or in vivo. The procedure of detection monitored alternations in subcellular nuclear such as the condensation process after proper destruction of the cell during the programmed cell death process. The high-frequency ultrasound technique shows a high scattering rate due to these intense alternations (approximately 25-50-fold) in apoptotic cells as compared to normal tissue cells. As a result, the apoptotic tissues show greatly brighter areas as compared to normal tissue. In the future, this noninvasive imaging technique will use to check the effect of anticancer treatment and chemotherapeutic agents in laboratory model systems and then in patients [103].

Another application of ultrasound technology is the successful detection of renal masses. According to research results, 86% carcinomas and 98% renal cysts were accurately determined among 111 patients by the ultrasound imaging technique. Ultrasound is a safe, simple, and cheap diagnostic tool to diagnose complex renal masses [104]. Ultrasound screening allows imaging the cartilage for checking instability, abnormal location of the femoral head inside the acetabulum, and developmental dysplasia in newborns [105]. A powerful low-frequency ultrasound system can also be used as a noninvasively drug delivery system. Many drugs and proteins having high molecular weight can be delivered easily with excessive permeability into human skin with the help of a low-frequency ultrasound modality. For example, insulin, erythropoietin, and interferon-gamma molecules are easily and safely delivered across human skin [106].

A novel molecular imaging technique known as molecular ultrasound has been used by researchers in the molecular biology field to monitor the alternation in the expression rate of molecular markers located on intravascular targets. Contrast agents used in the advanced molecular ultrasound imaging technology are mostly micro- or nanosized particles having ligands on the surface also known as microbubbles. Specific molecular markers are targeted by these microbubbles such as selectin, vascular cell adhesion molecule 1, and integrin. In this way, these agents lead to detect specific molecular markers on intravenous targets by gathering at that specific tissue site.

Molecular ultrasound has many advantages such as low-effective cost, high resolution, portable, noninvasiveness, absence of ionizing radiation, real-time imaging potential, and high availability. It has the potential for regular investigations of different abnormalities at the molecular level, such as inflammation, tumor angiogenesis, and thrombus. In addition, improvement is still required in the field of molecular ultrasound to design the novel targeting ligand to form a more effective contrast agent. In the future, advancements in molecular ultrasound imaging technology will play a clinical role with high sensitivity and accuracy for imaging complex abnormalities at the molecular level [107, 108].

## 21. Disadvantages of Medical Ultrasound

There are many useful applications of ultrasound in the medical field. But medical ultrasonography also had some side effects such as hormone change effect, breakage of chromosomes with very low frequency, chemical effects, and other health problems. It was examined that for 10-week gestation, chorionic gonadotropin hormone in humans increased after routine usage of ultrasound modality [109].

It was observed in an experiment that no chromosome damage occurred after diagnostic ultrasound exposure to human lymphocyte culture. But experimental results suggest that ultrasound can cause chromosome breakage with very low frequency [110]. Similarly, lots of experiments have been done to check fetal ultrasound safety. *In vivo* study demonstrates no major neurological defects, fetal growth problems, birth flaws, or childhood cancer caused by ultrasound imaging. But *in vitro* study demonstrates the possibility of some health problems that can occur due to diagnostic ultrasonography. For example, the effect of diagnostic ultrasound on the normal architecture of the mouse fibroblast cell with the production of fingerlike projections on the fine surface of the cell is demonstrated in Figure 15 [111].

Another disadvantage of an ultrasound system in the medical field is generating significant heat. When strong ultrasound waves migrate through the liquid environment, small cavities are produced, and these cavities expand, then collapse to each other, and generate heat. This heat-generating condition leads to create an unnecessary chemical environment [112]. Dyslexia, growth limitation, non-right handedness, and late speech-like effects are also examined after diagnostic ultrasound exposure. Continuous research is required to find the side effects of medical ultrasonography on human health [113].

## 22. Radiation Exposure Risk from Medical Imaging and Its Management

Radiological imaging by X-ray radiology, positron emission tomography (PET), single-photon emission computed tomography (SPECT), mammography, and computed tomography (CT) uses high-energy X-rays that leads to high radiation dose in some patients. Pregnant women and children are mostly affected by radiation exposure from radiological imaging. Possibility of cancer, genetic mutations, growth and developmental retardation in the fetus, and cardiovascular abnormalities can occur by the exposure to radiation after radiotherapy. Direct radiation exposure can cause hair loss, cataracts, skin redness, and skin damage. Radiation exposure risks can be reduced by making “National Guidelines” that aid the physician to manage their effects on patients.

Many online tools have been developed to enable physicians or technicians to record the calculation of radiation exposure from each radiological imaging technique. For this purpose, a Thermoluminescent dosimeter (TLD) is used to calculate radiation dose through different software depending on the modality being used such as Monte Carlo PENRADIO which is used for CT [114]. Magnetic resonance imaging (MRI) and ultrasound techniques are free from ionizing radiation. To minimize the risk, MRI and ultrasound can be used instead of radiological imaging techniques. Reduction in unnecessary computed tomography screening leads to the direct reduction of radiation exposure risks. Today, advanced and safe technologies are used that allow measuring signals with a low dose of radiation; e.g., low-dose computed tomography scanners permit less radiation exposure [115].

## 23. Advanced Machine Medical Image Analysis

4D medical imaging analysis is an advanced technology that is used in combination with different modalities such as 4D CT, 4D US, and 4D MRI. 4D CT is an excellent choice for radiation oncology, which is prone to motion artifacts. Similarly, 4D ultrasound is particularly useful in prenatal research. 4D flow MRI can help doctors diagnose and treat heart issues more precisely. For big data integration in medical imaging, researchers need to develop algorithms to store images by converting them into numerical format which will be helpful for physicians in diagnosis.

## 24. Artificial Intelligence in Medical Imaging

Machine learning and deep learning are branches of artificial intelligence (AI) that solves problems in medical imaging applications such computer-aided diagnosis, lesion segmentation, medical image analysis, image-guided treatment, annotation, and retrieval. AI assesses image quality, interprets image, and analyzes biomarkers, and finally, reporting is done. AI has impact on oncologic imaging. Lung cancer is one of the most prevalent and severe tumors in thoracic imaging. AI can assist in recognizing and classifying these nodules as benign or cancerous [116]. Machine learning focuses on pattern recognition. The traditional AI systems relied on preset engineering feature algorithms with specified parameters based on expert knowledge. Such features were intended to assess certain radiographic characteristics such as a tumor's 3D shape and intratumoral texture. Following that, a selection process ensures that only the most important features are used. The data is then fed into statistical machine learning models to find potential imaging-based biomarkers [117]. Deep learning algorithms learn by navigating the data space and by providing them with greater problem-solving capabilities. Convolutional neural networks (CNNs) are the most used deep learning architectural typologies in medical imaging today, even though many deep learning designs have been researched to handle diverse objectives [118].

## 25. Critical Analysis

Medical imaging often contains several techniques that are noninvasive to make images of different parts of the body. New imaging techniques such as computed tomography (CT), positron emission computed tomography (PET), magnetic resonance imaging (MRI), single-photon emission computed tomography (SPECT), ultrasound (US), and digital mammography reveal the internal anatomy and physiology of the body [2].

Advanced imaging technologies are used to diagnose various external as well as internal human illnesses that can also minimize diagnostic errors and produce novel and better information about the target object. There are benefits and risks to every imaging technique. Ultrasound is also employed in the medical field to look at the kidneys, heart, liver, blood vessels, and other organs of the body [95]. Computed tomography (CT) measures cancer and various abnormalities in the heart, abdomen, bone, and spinal cord with high resolution [33]. 3D ultrasound computed tomography (3D USCT) is a promising technology for the investigation of breast cancer [48]. PET is a powerful technique to visualize, characterize, and quantify the biological processes and pathological changes at the cellular and subcellular levels within a living body. The development of MRI is now employed to examine several musculoskeletal, neurologic problems, and cancer. It can be used for both soft and hard tissues [1]. Digital mammography is a rapid and computer-based modality. It is used for the diagnosis and screening of breast cancer [89].

Some imaging techniques, such as CT, PET, SPECT, and digital mammography using X-rays, lead to high ionizing radiation exposure risk in some patients. There are some management steps for minimizing the radiation exposure risks from imaging techniques [114]. The development in medical imaging techniques such as the use of PET/CT hybrid, SPECT/CT hybrid, 3D USCT, and simultaneous PET/MRI leads to an increase in our understanding of diseases and their treatment [84]. With advanced medical imaging techniques, detection of early-stage diseases is possible and then eventually aids patients to live longer and better lives. In the future, with mounting innovations and advancements in technology systems, the medical diagnostic field would become a field of regular measurement of various complex diseases and will provide healthcare solutions [1].

## Figures and Tables

**Figure 1:** CT scanner.

**Figure 2:** Distraction injury scanned by CT scan (showing damage occurrence at the 11^th^ and 12^th^ thoracic vertebrae).

**Figure 3:** An axial scan of a spinal injury by computed tomography (CT) at the 2^nd^ and 3^rd^ lumbar vertebrae.

**Figure 4:** (a) Femora undergo vQCT to determine BMD and macrostructure. (b) Ultradistal forearm undergoes CT to measure the structure of the trabecular complex network and its texture.

**Figure 5:** Microstructure of transiliac bone biopsies is determined to undergo 3D micro-CT of two postmenopausal women who have accomplished strontium ranelate therapy for 36 months: (a) strontium ranelate therapy; (b) placebo.

**Figure 6:** Images derived using a system known as GHNC (Gaussian Histogram Normalized Correlation). Lung images of a 73-year-old male IPF patient have been taken by computed tomography (CT). Light blue and yellow color, fibrosis; dark blue color, emphysema; pink color, normal; and light green color is indicated as ground-glass opacity.

**Figure 7:** Basic principle of PET scan: (1) a positive electron (positron) is emitted by radioactive decay of radioisotope, for example, carbon-11; (2) this positron hits an electron present in the tissue to be analyzed and emits two photons having low energy; (3) scintillation crystals are present in the PET camera to absorb this emitted photon with low energy; (4) the light is produced that is converted into another signal such as electrical signals used by the computer system to produce 3D images.

**Figure 8:** PET images of gene therapy in unilateral MPTP monkey as Parkinson's model: (a) image of normal dopamine production; (b) the image is representing autonomous dopamine MPTP-induced shortage (before gene therapy); (c) image of the restoration of dopamine production in the caudate and putamen (after gene therapy) [56].

**Figure 9:** Abnormal cerebral asymmetry in schizophrenia patients compared with control is shown by functional-MRI imaging technique.

**Figure 10:** Breast adenocarcinoma mouse model formed for the detection of lung metastases. (a) High-resolution hyperpolarized ^3^He MRI (HP ^3^He MRI) images were taken from the control mouse. Screening as normal ventilation forms of lungs. (b) After injection of LHRH-SPIONs, images were produced from human breast adenocarcinoma abnormal mouse (model), showing defects in the right lobe (under circles).

**Figure 11:** Dual-headed single-photon emission computed tomography (SPECT) system.

**Figure 12:** (a) The SPECT/CT scan of the knee joint shows clear articular cartilage. (b) The SPECT/CT arthrography image of the knee joint showing enhance the value of SPECT/CT screening.

**Figure 13:** (a) A healthy breast tissue mammogram recorded by digital mammogram; (b) the same breast tissue mammogram recorded by film mammography. White spots shown in the above images are deposits of calcium which can consider the mark of cancer when they form clusters.

**Figure 14:** (a) Hyphemia is due to injury; blood diffuses the anterior chamber of the eye. (b) Hyphemia scan image by Sonomed UBM.

**Figure 15:** Images of mouse fibroblast cell (a) normal smooth form and (b) abnormal cell in its rough shape. Due to the diagnostic ultrasound effect, fingerlike projections are produced on the smooth surface of the fibroblast cell.

## Data Availability

This is a review article. All data are taken from published research papers and available online.

## Abbreviations

AI: Artificial intelligence
BMD: Bone mineral density
CAT: Computed axial tomography
CT: Computed tomography
DCE-MRI: Dynamic contrast-enhanced magnetic resonance imaging
DFI: Disseminated fungal infection
DXA: Dual-energy X-ray absorptiometry
ECG: Electrocardiography
EEG: Electroencephalography
EIT: Electrical impedance tomography
EPI: Echo-planar imaging
ESI: Electrical source imaging
FDG: 2-[F-18] Fluoro-2-deoxy-D-glucose
FLT: 3-Deoxy-3-[F-18] fluorothymidine
fMRI: Functional MRI
fUS: Functional ultrasound
IPF: Idiopathic pulmonary fibrosis
LOC: Lab-on-a-chip
MEG: Magnetoencephalography
MPTP: 1-Methyl-4-phenyl-1,2,3,6-tetrahydropyridine
MRA: Magnetic resonance angiography
MRI: Magnetic resonance imaging
MRS: Magnetic resonance spectroscopy
NMR: Nuclear magnetic resonance
PEM: Positron emission mammography
PET: Positron emission tomography
PET-CT: PET and computed tomography
QCT: Quantitative CT
SIV: Simian immunodeficiency virus
SPECT: Single-photon emission computed tomography
SPION: Superparamagnetic iron oxide nanoparticles
TVS: Transvaginal ultrasound
UBM: Ultrasound biomicroscopy
3D USCT: Three-dimensional ultrasound computed tomography.
